The article "The Relationship between Urban Public Art and Regional Environment Based on Wireless Network Technology" was published in 2022. Journal: Comput Intell Neurosci.

# The Relationship between Urban Public Art and Regional Environment Based on Wireless Network Technology

**DOI:** 10.1155/2022/2872965

**Published:** 2022-05-19

**Authors:** Juan Li

**Affiliations:** College of Art and Design, Shanghai Normal University Tianhua College, Shanghai 201815, China

## Abstract

The relationship between urban public art and regional environment based on wireless network technology is studied. Combining domestic specific cases and referring to sociology, art, and design thinking, combing about the relationship between the city's public art and the regional environment, and further integration of its relationship components, at the same time, the planning study of Changning district, Shanghai, and the actual operation of the Shanghai Pudong International Airport, which incorporates the regional mesolevel background, are examples for case analysis. In reference cases and practical cases, they are deduced in sequence, starting from the environmental context of urban areas to the evolution model of public art. Moreover, the specific event background also constitutes a special opportunity period for the sudden growth of public art.

## 1. Introduction

There are two phases to the development of public art in contemporary China. The first is Hong Kong and Taiwan's earlier experience of absorbing the development of foreign public art and establishing independent institutions to promote the development of urban public art [1]. Furthermore, in recent years, major cities on the Mainland, such as Shenzhen, Beijing, and Shanghai, have actively conducted public art theoretical research and preliminary practical projects. Taiwan began researching and promoting public art such as fire and tea in the early 1990s, and in 1992, the “Regulations on Cultural and Arts Awards” were passed, defining the percentage of public art policies in Taiwan [2]. Every year since 1998, the competent authorities in charge of Taiwan's public art policy and implementation have compiled a “Yearbook of Public Art.” Simultaneously, he paid close attention to public art cultural studies, actively organized social resources, and published a large number of related works during Taiwan's development of public art. Hong Kong's public art has followed Taiwan's lead, and it has grown rapidly in the first decade of this century. The Hong Kong Arts Centre serves as the implementing agency for Hong Kong's “Public Art,” which was established in 2005 to promote the interaction of the arts, space, and the public. Its goal is to transform Hong Kong into a culturally vibrant metropolis. Interiorly, modern public art was enlightened in the late 1990s and has accelerated development in the last five years [3]. On the one hand, the advancement of public arts is linked to the advancement of the social environment, and on the other hand, it develops rapidly in the context of major historical events such as the Olympics and the World Expo [4].

## 2. State of the Art

The related topics of public art in China are based on the practical process of combining art with architecture and urban environment in the modernization after the reform and opening up. Whether it is the construction of murals or the development of urban sculptures, public art is involved in contemporary urban construction in various ways. In the face of vigorous development of practice, public art has lagged far behind in theory, breadth, and depth of research. Until the end of the 1980s, a group of well-known artists have conducted in-depth reflection on issues encountered in public art practice. The study of public art theory was first incorporated into the overall framework of contemporary social and cultural development [5]. Despite the fact that there are no monographs on regional environmental and public art relations studies in the publications related to public art, they provide a wealth of argumentation basis and can be roughly divided into four categories based on their contents: textbooks, thematic series, works, and doctoral student publications. Textbooks, whether they are monographs or other monographs, do not place a strong emphasis on problem exploration [6]. Its research aims to guide students in understanding the public consciousness in the social crowd through the concept and characteristics of public art and the design teaching of public art works so that students master a complete theoretical system and design method of public art design and then serve as a public art for students and the foundation of design ability and continuous research ability training [7]. As far as the research of this topic is concerned, these contents are the basic theory and case reference basis for the expansion of public art research. At the same time, from the compilation of a large number of public art related textbooks, it can be seen that public art is becoming a focus of training in domestic universities [8].

## 3. Methodology

### 3.1. Performance Analysis Algorithm Based on Key Chain Wireless Sensor Network Management Solution

It is possible that the above system will satisfy the security requirements of group key management in sensor networks [9–11], such as group key confidentiality, forward secrecy, and backward secrecy. We select *k* objects from *n* data objects to serve as the initial clustering centers and then group the other objects together based on how similar (or how far they are from these cluster centers) they are to these cluster centers (represented by the cluster center). Following that, the new cluster center value should be calculated (that is, the average of the objects in each cluster). This is repeated until the criteria function is no longer divergent. *K* objects *c*_1_, *c*_2_,…, *c*_*K*_ are randomly selected from the set of *n* objects {*x*_1_, *x*_2_,…, *x*_*n*_} as the center of the initial K sets of clusters. Taking *K* objects *c*_1_, *c*_2_,…, *c*_*K*_ as the center, each object is divided into the most similar collection. The specific division principle is as follows: if ‖*x*_*i*_ − *c*_*j*_‖ < ‖*x*_*i*_ − *c*_*m*_‖, *m*=1,2,…, *K*; *i*=1,2,…, *n* and *j* ≠ *m* divide *x*_*i*_ into the collection *C*_*j*_. We calculate the average of the objects in each newly-collected object collection: $\bar{x_{i}}=1/n_{i}\sum_{x\in C_{i}}x,i=1,2,\ldots ,K$, where *n*_*i*_ is the number of objects in the collection *C*_*i*_, so $C_{i}=\bar{x_{i}},i=1,2,\ldots ,K$. Calculation criterion function E is

(1) $$\begin{array}{c} E={\sum_{i=1}^{k}\sum_{x\in C_{i}}\left\|x-\bar{x_{i}}\right\|}^{2}. \end{array}$$

As a last resort, it is proceeded through step 2 until *E* does not appear to be changing any more. Because it is simple and rapid, the K-means algorithm [12] is a common solution for tackling the clustering problem. As a result, the approach is very scalable and efficient for processing big data sets, with a complexity of (n.k.t), where *n* is the total number of objects processed, *k* is the total number of clusters processed, and *t* is the total number of iterations processed. In the vast majority of circumstances, *k* + *n* and *t* + *n* are employed. The K-means method, on the other hand, has some shortcomings, including the following: because of the initial cluster center selection, it is possible that the K-means algorithm will converge to the local optimal solution before it is ready. When dealing with “noise” and outlier data, it is extremely sensitive, and even a small bit of it can have a significant impact on the average. The frequency distribution is defined as the distribution of the number of random events that occur in a certain number of trials (n trials in total). Variance is defined as the arithmetic mean of the square of dispersion. Specifically, the difference between each data in a group of data and the average of the group squared, summed, and divided by the number of data, represented by *σ*_*X*_^2^. Its definition formula is

(2) $$\begin{array}{c} \sigma_{X}^{2}=\frac{\sum {\left(X-\bar{X}\right)}^{2}}{N}. \end{array}$$

Among them, $X-\bar{X}$ represents the dispersion (that is, the difference between each data and the average), $\sum \left(X-\bar{X}\right)$ represents the sum of deviations, and N represents the total frequency. The standard deviation is the square root of the dispersion and the average square root. The square root of the variance, represented by *σ*_*X*_. Its definition formula is

(3) $$\begin{array}{c} \sigma_{X}=\sqrt{\frac{\sum {\left(X-\bar{X}\right)}^{2}}{N}}. \end{array}$$

The standard deviation and variance are two fundamental markers of variation between two groups. It is important to square and make the variance a positive number since the dispersion of each data point and the average is positive and negative, but the unit of data is also squared; therefore, the variance must be made positive. It is necessary to reopen the square in order to make the unit of difference quantity consistent with the original data. The skewness and kurtosis coefficients are statistics that are used to describe the characteristics of a data distribution. This has resulted in the inability to recover the group session key that existed prior to its inclusion. A steady-state distribution model of the Markov chain [13] is first provided in order to examine the computational overhead of the sensor nodes in the scheme, as well as the communication overhead between the key server and the nodes. A wireless sensor network's channel instability, which occurs when a node gets the key distribution message, might result in the loss of group key distribution message packets or the failure of authentication. These two events are deemed to have the same probability of occurring and can be treated as separate random events in this scenario. Because of this, it is simple to describe the key buffer status of each sensor node using a one-dimensional Markov chain, as seen in Figure 1. The state of the node $\alpha =\left(\sum {\left(X-\bar{X}\right)}^{3}/N\right)/\sigma_{X}^{3}$ represents the key buffer in the node, among other things.

When a key distribution message packet is lost or when a key update message event is successfully received [14], the node status is passed to the receiving node. If the frequency distribution is not normal, then the skewness coefficient and the kurtosis coefficient can be used to determine whether or not the distribution is normal. The following is the formula for determining the skewness coefficient when working with raw data:

(4) $$\begin{array}{c} \alpha =\frac{\sum {\left(X-\bar{X}\right)}^{3}/N}{\sigma_{X}^{3}}. \end{array}$$

Among them, *α* denotes the skewness coefficient, *X* denotes the original data, $\bar{X}$ denotes the average number, N denotes the total frequency, and *σ*_*X*_ denotes the standard deviation when *α*=0, indicating that the frequency distribution is in a symmetrical shape, which is in accordance with the normal distribution. When *α* > 0, the frequency distribution was positively skewed. When *α* < 0, it shows that the frequency distribution is negatively skewed. When using the raw data to calculate the kurtosis coefficient, the formula is

(5) $$\begin{array}{c} \beta =\frac{\sum {\left(X-\bar{X}\right)}^{4}/N}{\sigma_{X}^{4}}-3. \end{array}$$

Among them, *β* represents the kurtosis coefficient, *X* represents the original data, $\bar{X}$ represents the average number, N represents the total frequency, *σ*_*X*_ represents the standard deviation, and the distribution has a normal peak. When *β* > 0, the distribution showed a high narrow peak, at which time the average frequency around the ratio was large. The distribution pattern is highly narrow. The relationship between the urban public art and the regional environment is first considered in its entirety, and it is related to the development of the city. Different periods of urban appeal and development have a great influence on the degree of public art. The specific integration into the urban system, with the driving force as the reference point, reflects the relationship between the urban public art and the environment. There are mainly several modes: the government-planned policy promotes the development of the regional cultural image. The method of shaping public art as an image is concentrated in the municipal squares, streets, and parks. Here, the public art represents the regional environmental aesthetics business card and the values of regional culture; the specific events are temporary breakout points. At the emergence of public art sprawl in specific areas, such core areas of public art are mainly associated with specific space backgrounds such as the Olympic Park and Expo landscape belt; there is also a combination of specific cultural site backgrounds, such as universities and monumental parks, with cultural self-building and social communication as the driving force, from the inside out public art divergent setting.

### 3.2. The Constitutive Relationship between Public Art and Regional Environment

John Ayer and Rigoberto Tols have been creating public art in the South Bronx of New York for 13 years. This community is the poorest area in New York City. Violence, drug abuse, and home destruction are commonplace here. Aahan and Tols used the method of living to overturn and convert the most common residents of the community into a single statue, and part of it was permanently hung on the walls of the neighborhood. Residents are honored to be able to reappear in the works of the artist and have a new experience and understanding of their own life. Maybe art does not change the living habits of these people. However, they have changed the narrow and closed concept of space here, which has transformed the residents here towards openness. Obviously, what Ai Heng and Tols pursued was not the “artistic” effect of the work but the “social” effect; the problem they were trying to solve was not the issue of beautifying the city and beautifying the environment, but rather a social issue that was due to race. The artist advocated both the affirmation of cultural diversity and the spirit of tolerance for different cultures through this creative activity, as well as demonstrating profound humanistic care for society's bottom population. The civil society places a premium on the exercise of public rights. On the people's petition, the “oblique arc” sculpture on the welfare square in front of the Manhattan Federal Office Building mentioned in Chapter 2 was demolished. Designer Serra, on the other hand, filed a lawsuit in court, claiming that this was a violation. The First Amendment Act guarantees the right to freedom of expression. The Court of Appeal, on the other hand, recognized Serra's right to freedom of expression in principle while also arguing that Serra had already relinquished his right to freedom of expression when he turned the work over to the General Services Administration. The term “slope arc” refers to property rather than expression. Some important issues in public art are addressed in the “oblique arc” debate, such as the artist's right to express, public choice, and artistic expression under the constraints of property rights. This kind of property rights and public rights awareness not only drew attention in the United States several decades ago, but it is now increasingly influencing the realization of public art in today's domestic situation. Although most people were familiar with Shanghai Pudong International Airport's “Day at the Airport” series of scene sculptures, some passengers reported to the appropriate departments that one set of sculptures placed in chairs was occupying passengers. The rest, space, although the sculpture was not removed under the interpretation of coordination, it can be seen that the public is more sensitive to their own awareness of social rights, which also necessitates more careful consideration of space in the design and implementation process of public art. In China, the composition of human rights provides a more respected artistic experience for the general public. Citizens' spiritual needs are met first and foremost by contemporary urban public arts, which also promote the interaction of artistic needs. That is to say, artists use public works that are full of artistic appeal and cultural thinking to materialize social culture and public civilization in the form of public art. The public's cultural cognition is enhanced by people's cultural understanding, resulting in a socialized cultural artwork.

## 4. Result Analysis and Discussion

The relationship between public works of art and the environment is concerned, because the nature of the environment derived from the creation of public art is important, but this environment linkage does not need to be stereotyped as the inevitable requirements. The key is whether the installation of the work is to create a social significance for the public for the purpose of the aesthetic environment. As a result, this paper investigates and calculates using Shanghai as an example. Changning District has a permanent population of 690,600 people, 242,900 households, and an average household population of 2.49 people, according to the 2010 National Population Census results; daily residents are 334,600 men. There were 356,000 females, 21,400 more than males.

In addition to displaying basic population density data, these basic demographic data also provide some characteristics of the population environment in Changning District for the study of the project: the aging population tends to show a growing trend; the education level of the population is high; the population environment is diversified. The population has increased, the population of ethnic minorities has increased, and there is a relatively concentrated foreign population; the female population is high; the family size is small (Table 1). Therefore, focusing on the cultural life of the middle-aged and elderly people in the community as a background is a focus of public art; the protection of the local culture and the cultural context display will constitute a useful bridge between nonwoodland residents and communication; the scale of the family shows that the residents' attention to outdoor cultural life will be higher. As the East Hongqiao Business District has grown mature, its personnel education background should be higher than this average plan, which means that Hongqiao Business Centre as the energy of smart highlands will be more abundant; therefore, the artistic construction of this region also has a higher potential demand market. The promotion of public art as a means of promotion in high-quality population activity areas is also a choice to increase the satisfaction of residents in the area, and it is conducive to the formation of a virtuous cycle of comprehensive integration of talents. As is shown in Figure 2, Changning District is a comprehensive residential area with a wide range of areas and nature. From Xinli Residence to Garden House, from the grassroots community to the high-end villa area, the residential category and the nature of the residents are also distinct.

“Public art is the art of planning,” says the artist. One of the ways in which it differs from conventional contemporary art and contemporary art in general is that it incorporates conscious methodological knowledge into the design process. This is the first topic to look at the interaction between public art and the surrounding environment in depth. The fundamental conclusion is concerned with the logical chain of this relationship, and the continuation is concerned with the public art methodology that is employed in urban planning. In this article, the program's overall performance is assessed and reviewed. When compared to existing schemes, the key advantage of the suggested system is that group members can choose their own personal secret information without the need for the group administrator to communicate it through a secure channel. Each member of the group is simply required to keep the identity of the persons he or she chooses a secret from the others. When it comes to storage overhead, communication overhead, and security, the performance of this project compares favorably to that of analogous solutions, as shown in Table 1; *t* is the maximum number of collaborators that can be accommodated by the system, *m* is the total number of sessions that can be accommodated by the group life cycle, and *q* is a prime number that matches the cryptographic key specifications. The fundamental mechanism of the layer *μ* UTESLA protocol is depicted in Figure 3.

Our group members can choose their own personal secret information, as seen in Figure 2, and as a result, each group member only needs to keep a personal key of their choice throughout the self-healing key distribution process [15, 16]. It is necessary for scheme group members to maintain individual secret polynomial values that have been distributed by the group administrator, hence keeping the scheme's storage overhead to a minimum. After the parameter *p*_*L*_ changing to a different value, the graph of *E*[*N*^*H*^] as a function of the key buffer length *l* in Figure 4 can be seen in more detail. The average node update per key requires less computing overhead even when the channel packet loss rate is high (for example, *p*_*L*_ = 0.5), as illustrated in the diagram.

## 5. Conclusion

The results of public art reflected in different field backgrounds also have a symmetrical relationship with the environmental background. First of all, from the perspective of the city, the image language of the regional culture conveyed by the public art works depicts a certain aspect of the city image and is a label for the positioning of the city art; furthermore, from the specific regional environment, the public art often defines the vitality center of the region, infecting the public's sense of the environment with cultural cohesion; secondly, the positive energy that public art can transmit is also an important way of guiding social values. The exploration of the mode of public art also drives the corresponding discipline construction; essentially, the most important value of public art is the shaping of social cultural characters and the positive power of citizens' self-value recognition. The public experience is an important criterion for judging the value of public art in the environment. Public perception is a double-edged sword. On the one hand, public experience reflects the social value of public art. On the other hand, it is not enough for public perception. It may also hinder the realization of public art. Therefore, in the practice of public art and environment, we should pay attention to the value of the people's experience, but we should also do a good job of active cultural guidance.

## Figures and Tables

**Figure 1:** Diagram of sensor node state transitions.

**Figure 2:** Comparison of population living in different streets in Changning District.

**Figure 3:** Layered *μ* TESLA protocol basic mechanism.

**Figure 4:** Schematic diagram of calculation cost results of sensor nodes.

**Table 1:** Population characteristics of Changning district.

Classification	Population	Percentage of total population (%)	Compared to the previous census (%)	Ratio of the whole city (%)
65 and older	9.75 million	14.12	1.38	4
0–14 years old	4.80 million	6.95	4.24	1
All ethnic minorities	0.99 million	1.43	0.57	0.2
University level (college or above) population	25.73 million	37.26	18.04	1
Resident population	17.54 million	25.39	7.82	13

## Data Availability

The data used to support the findings of this study are available from the corresponding author upon request.
